The article "Exercise-induced mitochondrial p53 repairs mtDNA mutations in mutator mice" was retracted in 2021. Reason: duplicated images.

# Exercise-induced mitochondrial p53 repairs mtDNA mutations in mutator mice

**DOI:** 10.1186/s13395-016-0075-9

**Published:** 2016-01-31

**Authors:** Adeel Safdar, Konstantin Khrapko, James M. Flynn, Ayesha Saleem, Michael De Lisio, Adam P. W. Johnston, Yevgenya Kratysberg, Imtiaz A. Samjoo, Yu Kitaoka, Daniel I. Ogborn, Jonathan P. Little, Sandeep Raha, Gianni Parise, Mahmood Akhtar, Bart P. Hettinga, Glenn C. Rowe, Zoltan Arany, Tomas A. Prolla, Mark A. Tarnopolsky

**Affiliations:** 1 Department of Kinesiology, McMaster University, Hamilton, ON L8N 3Z5 Canada; 2 Department of Pediatrics, McMaster University, Hamilton, ON L8N 3Z5 Canada; 3 Department of Medicine, McMaster University, Hamilton, ON L8N 3Z5 Canada; 4 Department of Medical Sciences, McMaster University, Hamilton, ON L8N 3Z5 Canada; 5 Department of Medical Physics & Applied Radiation Sciences, McMaster University, Hamilton, ON L8N 3Z5 Canada; 6 Northeastern University, Boston, MA 02115 USA; 7 Buck Institute for Research on Aging, Novato, CA 94945 USA; 8 School of Health and Exercise Sciences, University of British Columbia Okanagan, Kelowna, BC V1V 1V7 Canada; 9 Division of Cardiovascular Disease, University of Alabama, Birmingham, AL 35294 USA; 10 Perelman School of Medicine, University of Pennsylvania, Philadelphia, PA 19104 USA; 11 Departments of Genetics, University of Wisconsin, Madison, WI 53706 USA; 12 Departments of Medical Genetics, University of Wisconsin, Madison, WI 53706 USA

**Keywords:** Skeletal muscle, Satellite cells, Endurance exercise, p53, Mitochondrial DNA mutations, Mutator mouse, Oxidative stress, Telomere, Apoptosis, Senescence

## Abstract

**Background:**

Human genetic disorders and transgenic mouse models have shown that mitochondrial DNA (mtDNA) mutations and telomere dysfunction instigate the aging process. Epidemiologically, exercise is associated with greater life expectancy and reduced risk of chronic diseases. While the beneficial effects of exercise are well established, the molecular mechanisms instigating these observations remain unclear.

**Results:**

Endurance exercise reduces mtDNA mutation burden, alleviates multisystem pathology, and increases lifespan of the mutator mice, with proofreading deficient mitochondrial polymerase gamma (POLG1). We report evidence for a POLG1-independent mtDNA repair pathway mediated by exercise, a surprising notion as POLG1 is canonically considered to be the sole mtDNA repair enzyme. Here, we show that the tumor suppressor protein p53 translocates to mitochondria and facilitates mtDNA mutation repair and mitochondrial biogenesis in response to endurance exercise. Indeed, in mutator mice with muscle-specific deletion of p53, exercise failed to prevent mtDNA mutations, induce mitochondrial biogenesis, preserve mitochondrial morphology, reverse sarcopenia, or mitigate premature mortality.

The article "Exercise-induced mitochondrial p53 repairs mtDNA mutations in mutator mice" was retracted in 2021. Reason: duplicated images.

**Conclusions:**

Our data establish a new role for p53 in exercise-mediated maintenance of the mtDNA genome and present mitochondrially targeted p53 as a novel therapeutic modality for diseases of mitochondrial etiology.

**Electronic supplementary material:**

The online version of this article (doi:10.1186/s13395-016-0075-9) contains supplementary material, which is available to authorized users.

## Background

The universality of the aging phenomenon has evoked great interest in unveiling regenerative remedies and rejuvenation medicine designed to evade molecular instigators of mammalian aging. Molecular investigations of age-related pathologies implicate mitochondrial DNA (mtDNA) mutations as one of the primary instigators driving multisystem degeneration, stress intolerance, and energy deficits [1]. It is intuitive to assume that the de novo mtDNA mutations observed during aging are due to accumulated, unrepaired oxidative damage, but some evidence actually suggests that mtDNA replication errors may be the more important culprit [2]. The demonstration that multiple aspects of aging are accelerated in mutator mice harboring error-prone mitochondrial polymerase gamma provides support for the causal role of mtDNA replication errors in instigating mammalian aging [3, 4]. Similar phenotypes have also been reported in telomerase-deficient mice [5], where telomere dysfunction is associated with impaired mitochondrial biogenesis and metabolic failure resulting in progressive tissue atrophy, stem cell depletion, organ system failure, and impaired tissue injury responses as seen with aging [5]. Indeed, epidemiological studies have correlated decreased telomere length in peripheral blood leukocytes, with higher mortality rates in individuals more than 60 years old [6]. Furthermore, a recent study in centenarians and their offspring found a positive link between telomere length and longevity; in particular, those with longer telomeres had an overall improved health profile, with decreased incidence of age-associated diseases, better cognitive function, and improved lipid profiles relative to controls [7].

The epidemic emergence of modern chronic diseases largely stems from the adoption of a sedentary lifestyle and excess energy intake [8]. There is incontrovertible evidence that endurance exercise extends life expectancy and reduces the risk of chronic diseases in both rodents and humans [9, 10]. We have previously shown that endurance exercise effectively rescued progeroid aging in mutator mice concomitant with a reduction in mtDNA mutations, despite an inherent defect in mitochondrial polymerase gamma (POLG1) proofreading function [11]. Exercise has also been shown to increase telomerase activity and reduce senescence markers [12]. These findings suggest a link between exercise-mediated metabolic adaptations and genomic (nuclear and mitochondrial) stability; however, the identity of this metabolic link remains unknown. In this study, we have utilized PolG mice to investigate the mitochondrial-telomere dysfunction axis in the context of progeroid aging, and to elucidate how exercise counteracts mitochondrial dysfunction and mtDNA mutation burden through mitochondrial localization of the tumor suppressor protein p53.

The article "Exercise-induced mitochondrial p53 repairs mtDNA mutations in mutator mice" was retracted in 2021. Reason: duplicated images.

## Methods

### Mice breeding

Heterozygous mice (C57Bl/6J, *PolgA* ^*+/D257A*^) for the mitochondrial polymerase gamma knock-in mutation were a kind gift from Dr. Tomas A. Prolla, University of Wisconsin-Madison, USA [4]. We generated homozygous knock-in mtDNA mutator mice (PolG; *PolgA* ^*D257A/D257A*^) and littermate wild-type (WT; *PolgA* ^*+/+*^) from heterozygous mice-derived colony maintained at the McMaster University Central Animal Facility as previously described [11]. Muscle-specific p53 knock-out mice (p53 MKO) were bred by crossing p53 flox mice (*Trp53* ^*tm1Brn*^/J) with muscle-creatine kinase Cre recombinase mice (Tg(Ckmm-cre)5Khn/J) purchased from Jackson Laboratories. We generated genetically modified homozygous knock-in mtDNA mutator mice with muscle-specific p53 knockout (PolG-p53 MKO), by crossing heterozygous mice (*PolgA* ^*+/D257A*^) with p53 MKO mice. During breeding, all animals were housed three to five per cage in a 12-h light/dark cycle and were fed ad libitum (Harlan-Teklad 8640 22/5 rodent diet) after weaning. The presence of the polymerase gamma homozygous knock-in mutation was confirmed as previously described [4].

### Endurance exercise protocol

Endurance exercise protocol and tissue harvesting was carried out, as previously described, using an independent cohort of mice [11]. Briefly, at 3 months of age, mice were housed individually in micro-isolator cages in a temperature- and humidity-controlled room and maintained on a 12-h light–dark cycle with food and water ad libitum [13]. PolG mice and PolG-p53 MKO mice were randomly assigned to sedentary (PolG-SED or PolG-p53 MKO-SED) or forced-endurance (PolG-END or PolG-p53 MKO-END) exercise groups (*n* = 5–20/group; ♀ = ♂). None of the mice had been previously subjected to a structured exercise regiment. One week of pre-training was allowed to acclimatize mice in endurance exercise groups to the treadmill. Mice in endurance exercise groups were subjected to forced treadmill exercise (Eco 3/6 treadmill; Columbus Instruments, Columbus, Ohio) three times per week at 15 m/min for 45 min for 6 months. A 5-min warm-up and cool-down at 8 m/min were also included. PolG mice were age- and sex-matched with sedentary littermate WT mice (*n* = 20; ♀ = ♂), which served as controls for the study to assess if endurance exercise intervention can molecularly bring PolG mice to normalcy. At 8 months of age, animals were euthanized and tissues were collected for molecular analyses. The study was approved by the McMaster University Animal Research and Ethics Board under the global Animal Utilization Protocol # 12-03-09, and the experimental protocol strictly followed guidelines put forth by the Canadian Council of Animal Care.

The article "Exercise-induced mitochondrial p53 repairs mtDNA mutations in mutator mice" was retracted in 2021. Reason: duplicated images.

### Endurance stress test

The mice were subjected to four separate endurance stress tests over to indirectly assess improvements in aerobic capacity with exercise as previously described [11]. Briefly, animals from all groups were placed in individual lanes on the treadmill and allowed to acclimatize for 30 min to eliminate any confounding effects due to stress or anxiety related to a new environment. The test began with a 5-min warm-up session at 8 m/min, followed by +1 m/min increase in speed every 2 min until the mouse reached exhaustion. A low-intensity electrically stimulus was provided to ensure compliance. Time to exhaustion (min) was recorded when the mouse sat at the lower end of the treadmill, near a shock bar, for >10 s and was unresponsive to further stimulation to continue running.

### Survival analysis

An independent cohort of animals from all groups was used to carry out survival analyses as previously described [11], and Kaplan–Meier survival curves were calculated using GraphPad Prism 4.0.

### Tissue harvesting

Tissues were collected at the time of euthanasia as previously described [11]. Immediately following cervical dislocation, the chest cavity was exposed and the heart was removed rapidly, followed by the skeletal muscle (*quadriceps femoris*). The skeletal muscle (*quadriceps femoris*, *tibialis anterior*, and *soleus*) and heart were either (i) collected in RNase-free cryovials, immediately immersed in liquid nitrogen, and stored at −80 °C for later analysis of DNA, RNA, protein, and enzyme activity or (ii) immediately rinsed with phosphate buffer saline (PBS) and used for skeletal muscle and heart mitochondrial and nuclear fractionations.

### Hematopoietic stem and progenitor cell isolation

Mouse hematopoietic stem and progenitor cells (HSC) were isolated according to the method of Ema et al. with minor modifications [14]. Marrow was flushed from the femur and tibia using a 25-g needle, passed through a 50-μm sieve and counted with a hemocytometer. Cells were incubated with primary antibodies for 90 min at 4 °C followed by 20 min incubation in the appropriate secondary antibody at 4 °C. Lineage negative, and Sca-1 and c-Kit positive (LSK) population enriched for stem cells were sorted using the EPICS ALTRA™ fluorescence-activated cell sorter (Beckman Coulter, Mississauga, ON) with gating strategies established using single-stained controls. The following antibodies were used: lineage panel (BD Pharmingen™, Mississauga, ON), anti-mouse Sca-1 Clone: E13-161.7 (BD Pharmingen™, Mississauga, ON), anti-mouse c-Kit Clone: 2B8 (eBioscience, San Diego, CA), and streptavidin (BioSource, Burlington, ON).

The article "Exercise-induced mitochondrial p53 repairs mtDNA mutations in mutator mice" was retracted in 2021. Reason: duplicated images.

### Satellite cell isolation

Primary skeletal muscle satellite cells (SC) were isolated from WT, PolG-SED, and PolG-END mice using the methods described previously [15] and subsequently purified by fluorescence-activated cell sorting. Briefly, the hind limb skeletal muscles were carefully dissected, cleaned of fat and washed in cold PBS. Cells were released by mulching the tissue with scissors and incubation in a collagenase/dispase solution three times, 12 min each, at 37 °C with further mechanical disruption using a pipette between incubations. Following passage through 70 and 30 μm filters, cells were stained using primary antibody to c-met conjugated to PE (1:200, eBioscience, San Diego, CA) and subjected to FACS sorting (EPICS ALTRA™, Beckman Coulter, Mississauga, ON). SC were pelleted in RNase-free cryovials, immediately immersed in liquid nitrogen, and stored at −80 °C for later analyses.

### Mouse embryonic fibroblast isolation and reporter assay

Mouse embryonic fibroblasts (MEFs) were generated using standard techniques from WT (p53^+/+^) and p53 knockout (KO) mice (p53^−/−^). Cell used in the experiments were from passages 4–5. Promoter sequence for PGC-1α was amplified by PCR from mouse muscle genomic DNA and cloned into the pGL4 luciferase reporter vector (Promega, Madison, WI). The pG13-luc plasmid containing 13 copies of a synthetic p53 DNA binding site was used as a positive control (which has been comprehensively characterized in Jackson et al., 2001 and Kern et al., 1991). A GFP expressing plasmid was used to normalize transfection efficiency. p53^+/+^ and p53^−/−^ MEFs were transfected (Lipofectamine 2000, Invitrogen, Burlington, ON) with either empty pGL4, pG13-luc (positive control), or pGL4-PGC-1α vectors. p53 transcriptional activity was measured using Bright-Glo™ luciferase reporter assay system (Promega, Madison, WI).

### Total RNA isolation from skeletal muscle and heart

Total RNA was isolated from ~25 mg of the skeletal muscle (*quadriceps femoris*) and heart using the Qiagen total RNA isolation kit (Qiagen, Mississauga, ON) [11, 13]. RNA samples were treated with RNase-free DNase on Qiagen spin-columns (Qiagen, Mississauga, ON) to remove DNA contamination. RNA integrity and concentration were assessed using the Agilent 2100 Bioanalyzer (Agilent Technologies, Palo Alto, CA) [13]. The average RIN (RNA integrity number) value for all samples was 9.64 ± 0.20 (scale 1–10), ensuring a high quality of isolated RNA.

The article "Exercise-induced mitochondrial p53 repairs mtDNA mutations in mutator mice" was retracted in 2021. Reason: duplicated images.

### RNA, DNA, and protein isolation from HSC and SC

Total RNA, DNA, and protein were isolated from HSC and SC using the Qiagen AllPrep DNA/RNA Mini Kit (Qiagen, Mississauga, ON) according to the manufacturer’s instructions.

### Microarray analysis

Total RNA was extracted from skeletal muscle (*quadriceps femoris*) using the Qiagen RNeasy Micro kit (Qiagen, Mississauga, ON) and processed on Qiagen’s QIAcube (Qiagen, Mississauga, ON) using the standard manufacturer’s protocol. The samples were then checked for quality using Nanodrop 2000 (Thermo Scientific, Wilmington, DE) and Agilent 2100 Bioanalyzer (Agilent Technologies, Palo Alto, CA). TransPlex Whole Transcriptome Amplification kit (Sigma-Aldrich^®^, Oakville, ON) was used to amplify complementary (cDNA) from the muscle RNA samples according to the manufacturer’s instructions. Samples were amplified for 25 cycles using the recommended cycling parameters. All samples were subsequently purified using Qiagen’s QIAquick PCR Purification kit (Qiagen, Mississauga, ON) and processed on Qiagen’s QIAcube (Qiagen, Mississauga, ON) using the standard “Cleanup QIAquick PCR for amplification reactions” (Version 4) protocol. Samples were purified and examined using Nanodrop 2000 (Thermo Scientific, Wilmington, DE) and Agilent 2100 Bioanalyzer DNA 7500 chip (Agilent Technologies, Palo Alto, CA) to ensure proper yield and quality of amplification. To perform the microarray hybridization, 2 μg of cDNA from each sample was labeled using NimbleGen’s One Color Labeling kit (Cat.# 05223555001; Roche NimbleGen Inc., Madison, WI) according to the manufacturer’s protocol. Five micrograms of Cy3 labeled samples were hybridized to *Mus musculus* 12x135k, NimbleGen Gene Expression Arrays (Cat.# 05543797001; Roche NimbleGen Inc., Madison, WI), washed, and scanned according to manufacturer’s protocol. NimbleGen gene expression arrays were scanned using an Axon GenePix 4200A scanner (Molecular Devices Inc., Downingtown, PA) with settings of 100 POW and 300–350 photomultiplier (PMT). Pair files were generated for each array using NimbleScan software (Roche NimbleGen Inc., Madison, WI). Resulting array data was analyzed with Bioconductor software (Bioconductor, Seattle, WA) in which the data were normalized and tested for significantly differentially expressed genes which were assessed based upon a 5 % false discovery rate (FDR). The gene array data reported here is deposited in Gene Expression Omnibus (Accession Number: GSE75869) public functional genomics data repository. The resulting data were input into Ingenuity Pathway Analysis (Ingenuity^®^ Systems, Redwood City, CA) to determine the over-represented gene categories using strict association. The normalized expression in these categories was plotted in a heat map using R script and Bioconductor software (Bioconductor, Seattle, WA).

The article "Exercise-induced mitochondrial p53 repairs mtDNA mutations in mutator mice" was retracted in 2021. Reason: duplicated images.

### Real-time quantitative PCR

The messenger RNA (mRNA) expression of peroxisome proliferator-activated receptor gamma co-activator 1 alpha (PGC-1α), mitochondrial transcription factor A (TFAM), estrogen-related receptor alpha (ERRα), 5-aminolevulinate synthase (ALAS), cytochrome *c* oxidase subunit-I (COX-I), cytochrome *c* oxidase subunit-IV (COX-IV), complex I NADH dehydrogenase subunit 1 (ND1), complex V subunit ATPase 6 (ATPase 6), cyclin-dependent kinase inhibitor 1A (p21^WAF1^), cyclin-dependent kinase inhibitor 2A (p16^INK4A^), and growth arrest and DNA-damage-inducible beta (GADD45B) were quantified using 7300 Real-time PCR System (Applied Biosystems Inc., Foster City, CA) and SYBR^®^ Green chemistry (PerfeC_T_a SYBR^®^ Green Supermix, ROX, Quanta BioSciences, Gaithersburg, MD) as previously described [11, 13]. First-strand cDNA synthesis from 1 μg of total RNA was performed with random primers using a high-capacity cDNA reverse transcription kit (Applied Biosystems Inc., Foster City, CA) [11]. Forward and reverse primers for the aforementioned genes (Additional file 1: Table S2) were designed based on sequences available in GenBank using the online MIT Primer 3 designer software (developed at Whitehead Institute and Howard Hughes Medical Institute by Steve Rozen and Helen Skaletsky) and were confirmed for specificity using the basic local alignment search tool. β-2 microglobulin was used as a control house-keeping gene, as its expression was not affected with the experimental intervention (data not shown). All samples were run in duplicate simultaneously with a negative control which contained no cDNA. Melting point dissociation curves generated by the instrument were used to confirm the specificity of the amplified product.

### Tissue total DNA isolation

Total DNA (genomic and mtDNA) was isolated from ~15 mg of the skeletal muscle (*soleus*) and heart using the QIAamp DNA Mini kit (Qiagen, Mississauga, ON) [11, 16]. DNA samples were treated with RNase (Fermentas, Mississauga, ON) to remove RNA contamination. DNA concentration and quality were assessed using Nanodrop 2000 (Thermo Scientific, Wilmington, DE).

The article "Exercise-induced mitochondrial p53 repairs mtDNA mutations in mutator mice" was retracted in 2021. Reason: duplicated images.

### mtDNA copy number analysis

Mitochondrial DNA copy number, relative to the diploid chromosomal DNA content, was quantitatively analyzed from the skeletal muscle (*soleus*), heart, primary hematopoietic stem cells, primary satellite cells, and primary fibroblasts using ABI 7300 real-time PCR (Applied Biosystems, CA) [11, 16]. Primers were designed around COX-II region of the mitochondrial genome (Additional file 1: Table S2). Nuclear β-globin gene was used as a housekeeping gene (Additional file 1: Table S2).

### Average telomere length

Average telomere length was measured in heart, primary hematopoietic stem cells, and primary satellite cell genomic DNA using a real-time quantitative PCR method as previously described [17]. The premise of this assay is to measure an average telomere length ratio by quantifying telomeric DNA with specially designed primer sequences and dividing that amount by the quantity of a single-copy gene [17]. All samples were run using a 7300 Real-time PCR System (Applied Biosystems Inc., Foster City, CA) and SYBR^®^ Green chemistry (PerfeC_T_a SYBR^®^ Green Supermix, ROX, Quanta BioSciences, Gaithersburg, MD). A single-copy gene, 36B4, which encodes for the acidic ribosomal phosphoprotein PO, was used as a control for amplification for every sample performed [17, 18]. Each PCR reaction for the telomere and 36B4 included 12.5 μL of 1x SYBR^®^ Green master mix (PerfeC_T_a SYBR^®^ Green Supermix, ROX, Quanta BioSciences, Gaithersburg, MD), 300 nM each of the forward and reverse telomere or 36B4 primers (Additional file 1: Table S2), 20 ng genomic DNA, and enough DNase/RNase-free H_2_O (Applied Biosystems Inc., Foster City, CA) to yield a 25-μL reaction. Cycling conditions for telomere are as follows: 95 °C for 10 min followed by 30 cycles of data collection at 95 °C for 15 s and a 56 °C anneal-extend step for 1 min. Cycling conditions for 36B4 are as follows: 95 °C for 10 min followed by 35 cycles of data collection at 95 °C for 15 s, with 52 °C annealing for 20 s, followed by extension at 72 °C for 30. Each sample was analyzed in duplicate, and the ratio of telomere:36B4 was calculated. The average of these ratios was reported as the average telomere length ratio (ATLR).

### Whole tissue lysate

Total protein was extracted from tissue samples as previously described [11]. Briefly, ~30 mg of the skeletal muscle (*quadriceps femoris*) and heart were homogenized on ice in a 2-mL Wheaton glass homogenizer (Fisher Scientific, Ottawa, ON) with 25 volumes of phosphate homogenization buffer [50 mM KPi, 5 mM EDTA, 0.5 mM DTT, 1.15 % KCl supplemented with a Complete Mini, ETDA-free protease inhibitor cocktail tablet and a PhosSTOP, phosphatase inhibitor cocktail tablet (Roche Applied Science, Mannhein, Germany) per 10 mL of buffer]. The lysate was centrifuged at 600*g* for 15 min at 4 °C to pellet cellular debris. The supernatant was aliquoted, snap frozen in liquid nitrogen, and stored at −80 °C until further analysis.

The article "Exercise-induced mitochondrial p53 repairs mtDNA mutations in mutator mice" was retracted in 2021. Reason: duplicated images.

### Nuclear fractionation

Nuclear fractions were prepared from 40 mg of the freshly obtained skeletal muscle (*quadriceps femoris*), heart, primary satellite cells, and primary fibroblasts using a commercially available nuclear extraction kit (Pierce NE-PER^®^, Rockford, IL) as previously described [11, 16]. Briefly, samples were homogenized in CER-I buffer containing protease inhibitor cocktail Complete, ETDA-free (Roche Applied Science, Mannheim, Germany) using an electronic homogenizer (Pro 250, Pro Scientific, Oxford, CT, USA). Pellets containing nuclei were obtained by centrifugation at 16,000*g* for 10 min at 4 °C and were subsequently washed four times in PBS to remove cytosolic contaminating proteins. Nuclear proteins were extracted in NER buffer supplemented with protease inhibitors [11]. Enrichment and purity of nuclear fractions were confirmed by the abundance of nuclear histone H2B and absence of the cytosolic protein lactate dehydrogenase in Western blot analyses as previously shown by our group [16].

### Chromatin immunoprecipitation assay

Chromatin immunoprecipitation (ChIP) assay was performed using an EZ-ChIP™ kit (Millipore, Billerica, MA) as previously described [11]. Twenty-milligram piece of the *quadriceps femoris* muscle was cross-linked in 5 mL of phosphate-buffered saline containing 1 % formaldehyde for 10 min at room temperature. One milliliter of 10X glycine was added to stop fixation. Muscles were then homogenized in 1 mL of SDS lysis buffer supplemented with protease inhibitor cocktail Complete, ETDA-free (Roche Applied Science, Mannheim, Germany). Chromatin was sheared by sonicating each sample on ice using a Branson Digital Sonifier^®^ S-450D (output 20 %, 4 times for 20 s, with a 20-s pause each time; Branson Ultrasonics Corporation, Danbury, CT). Following centrifugation at 10,000×*g* at 4 °C for 10 min, the supernatant containing 1 mg of protein was diluted to 1 mL with dilution buffer. Ten micrograms of anti-p53 (FL-393) antibody (Santa Cruz Biotechnology Inc., Santa Cruz, CA) was added per sample and incubated overnight at 4 °C. Anti-IgG antibody was used as a non-specific control. Sixty microliters of protein G-agarose was added, and the sample was mixed for 1 h at 4 °C with rotation. Precipitated complexes were eluted in 100 μL of elution buffer, and cross-linking was reversed by the addition of 8 μL of 5 M NaCl per sample followed by incubation at 65 °C for 10 h. Co-immunoprecipitated DNA was purified according to the manufacturer’s instructions. Primers were designed to amplify the p53 binding regions (−564 and −954) of the PGC-1α promoter (Additional file 1: Table S2). The amount of PGC-1α promoter immunoprecipitated with p53 was quantified using the 7300 Real-time PCR System (Applied Biosystems Inc., Foster City, CA) and SYBR^®^ Green chemistry (PerfeC_T_a SYBR^®^ Green Supermix, ROX, Quanta BioSciences, Gaithersburg, MD). Purified DNA from the input sample that did not undergo immunoprecipitation was PCR-amplified using of β-globin primers (Additional file 1: Table S2) and was used to normalize signals from ChIP assays.

The article "Exercise-induced mitochondrial p53 repairs mtDNA mutations in mutator mice" was retracted in 2021. Reason: duplicated images.

### Mitochondrial fractionation

Mitochondrial fractions were isolated using differential centrifugation as previously outlined [11]. Briefly, the skeletal muscle (*quadriceps femoris* and *tibialis anterior*), heart, primary satellite cells, and primary fibroblasts were finely minced and homogenized on ice in 1:10 (wt/vol) ice-cold isolation buffer A (10 mM sucrose, 10 mM Tris/HCl, 50 mM KCl, and 1 mM EDTA, and 0.2 % fatty acid-free BSA, pH 7.4, supplemented with protease inhibitor cocktail Complete, ETDA-free [Roche Applied Science, Mannheim, Germany]) using a Potter-Elvehjem glass homogenizer. The resulting homogenates were centrifuged for 15 min at 700*g*, and the subsequent supernatants were centrifuged for 20 min at 12,000*g*. The mitochondrial pellets from 12,000*g* spin were washed and then re-suspended in a small volume of ice-cold isolation buffer B (10 mM sucrose, 0.1 mM EGTA/Tris, and 10 M Tris/HCl, pH 7.4, supplemented with protease inhibitor cocktail Complete, ETDA-free [Roche Applied Science, Mannheim, Germany]). All centrifugation steps were carried out at 4 °C. The mitochondrial pellets were immediately frozen at −80 °C for further biochemical analyses. Enrichment and purity of mitochondrial fractions were confirmed by the abundance of mitochondrial cytochrome *c* oxidase subunit IV protein and absence of the nuclear histone H2B and the cytosolic protein lactate dehydrogenase in Western blot analyses as previously shown by our group [16].

### Mitochondrial co-immunoprecipitation assay

Mitochondrial co-immunoprecipitation assay was performed on isolated mitochondrial fractions using Pierce Co-Immunoprecipitation Kit (Pierce, Rockford, IL) as previously described [16]. Briefly, mitochondrial fractions were homogenized in lysis buffer (0.025 M Tris, 0.15 M NaCl, 0.001 M EDTA, 1 % NP-40, 5 % glycerol, pH 7.4) supplemented with protease inhibitor cocktail Complete, ETDA-free (Roche Applied Science, Mannheim, Germany). Two milligrams of mitochondrial fraction was pre-cleared by incubation with 100 μL of control agarose resin to minimize non-specific binding. Forty micrograms of anti-p53 (FL-393) antibody (Santa Cruz Biotechnology Inc., Santa Cruz, CA) was covalently coupled onto an amine-reactive resin. The pre-cleared lysates were subsequently incubated with antibody-coupled beads overnight at 4 °C. Co-immunoprecipitates were collected by centrifugation, boiled in 50 μL of Laemmli sample buffer, and used for immunoblot analysis for POLG1 (a kind gift of Dr. William C. Copeland, National Institutes of Health) or anti-Tfam (sc23588, A-17; Santa Cruz Biotechnology Inc., Santa Cruz, CA) antibody. Anti-IgG antibodies were used as a non-specific control.

The article "Exercise-induced mitochondrial p53 repairs mtDNA mutations in mutator mice" was retracted in 2021. Reason: duplicated images.

### mtDNA immunoprecipitation assay

mtDNA immunoprecipitation was performed on skeletal muscle mitochondrial fraction that was cross-linked and sonicated as previously described [16, 19]. One milligram of mitochondrial fraction was pre-cleared in 25 % *v*/*v* pre-clearing matrix F (Santa Cruz Biotechnology, Santa Cruz, CA) overnight at 4 °C. The supernatant was then incubated with 20 μg of anti-p53 (FL-393) antibody (Santa Cruz Biotechnology Inc., Santa Cruz, CA) and ExactaCruz™ F matrix (Santa Cruz Biotechnology, Santa Cruz, CA) [20] with mixing by end-over-end inversion overnight at 4 °C in the presence of 5 μg of shared salmon sperm DNA (Sigma-Aldrich^®^, Oakville, ON) to reduce non-specific DNA-bead interactions. Anti-IgG antibodies were used as a non-specific control. The matrix was centrifuged at 16,000*g* for 30 s, and the pellet matrix-immune complex precipitate was washed four times under stringent conditions (50 mM Tris-HCl, pH 7.4, 500 mM NaCl, 2 mM EDTA) and incubated overnight at 65 °C in the presence of 1 % SDS for cross-linking reversion. DNA was extracted from supernatants using the QIAamp DNA Mini kit (Qiagen, Mississauga, ON) according to the manufacturer’s instructions. mtDNA COX-II and cytochrome *b* regions (Additional file 1: Table S2) were quantified using 7300 Real-time PCR System (Applied Biosystems Inc., Foster City, CA) and SYBR^®^ Green chemistry (PerfeC_T_a SYBR^®^ Green Supermix, ROX, Quanta BioSciences, Gaithersburg, MD), as previously described [16].

### Western blotting and markers of oxidative damage

Protein concentrations of whole tissue lysates, and mitochondrial and nuclear fractions were determined using a commercial assay (BCA Protein Assay, Pierce, Rockford, IL). Proteins were resolved on 10 or 12.5 % SDS-PAGE gels depending on the molecular weight of the protein of interest. The gels were transferred onto Hybond^®^ ECL nitrocellulose membranes (Amersham, Piscataway, NJ) and immunoblotted using the following commercially available primary antibodies: MitoProfile^®^ Total OXPHOS Rodent cocktail (MS604) antibody (MitoSciences, Eugene, OR); anti-PGC-1α (2178), anti-VDAC (4866), and anti-α/β-tubulin (2148) antibodies (Cell Signaling Technology, Denver, MA); anti-p53 (MABE283-PAb421) antibody (EMD Millipore); anti-Tfam (sc-23588) and anti-NRF-1 (sc-33771) antibodies (Santa Cruz Biotechnology Inc., Santa Cruz, CA); anti-POLG1 antibody (a kind gift of Dr. William C. Copeland, National Institutes of Health, USA); anti-citrate synthase antibody (a kind gift of Dr. Brian H. Robinson, The Hospital for Sick Children, Canada); anti-4-HNE (ab48506), anti-SOD2 (ab13533), anti-catalase (ab1877), and anti-p21^WAF1^ (ab7960) antibodies (Abcam, Cambridge, MA); anti-Pax7 (Developmental Studies Hybridoma Bank, University of Iowa, Iowa City, IO); and anti-ERRα (EPR46Y) and anti-actin (NB600-535) antibodies (Novus Biologicals, Littleton, CO) [11, 16]. The carbonylated protein content in whole tissue lysates and mitochondrial fractions was quantified by Western blot using OxyBlot Protein Detection kit (S7150; Millipore, Bedford, MA) as per manufacturer’s instructions. All antibodies were used at 1:1000 dilution, except for anti-actin (1:10,000). Membranes were then incubated with the appropriate anti-mouse or anti-rabbit horse radish peroxidase-linked secondary antibody (1:10,000) and visualized by enhanced chemiluminescence detection reagent (Amersham, Piscataway, NJ). Relative intensities of the protein bands were digitally quantified by using NIH Image J, version 1.37, analysis software (Scion Image, NIH).

The article "Exercise-induced mitochondrial p53 repairs mtDNA mutations in mutator mice" was retracted in 2021. Reason: duplicated images.

### ROS assay

Mitochondrial H_2_O_2_ production was measured using the Amplex^®^ Red Hydrogen Peroxide assay (A22188; Invitrogen, Burlington, ON) as per manufacturer’s instructions. Briefly, 40 μg of mitochondrial fraction was diluted in 50 μL reaction buffer (125 mM KCl, 10 mM HEPES, 5 mM MgCl_2_, 2 mM K_2_HPO_4_, pH 7.44) to determine mitochondrial respiratory chain complex I (5 mM pyruvate/malate) or complex II (5 mM succinate) driven H_2_O_2_ production with and without inhibitors (0.5 μM rotenone, complex I inhibitor, and 0.5 μM antimycin A, complex III inhibitor). Mitochondrial H_2_O_2_ production was measured after the addition of 50 μL of reaction buffer containing horseradish peroxidase and Amplex^®^ Red. Fluorescence was followed at an excitation wavelength of 545 nm and an emission wavelength of 590 nm for 5 min using fluorescence microplate reader (Tecan Safire, MTX Lab Systems, Inc., Vienna, VA). The slope of the increase in fluorescence is converted to the rate of H_2_O_2_ production with a standard curve. All of the assays were performed at 25 °C. The results are expressed as pmoles.min^−1^.mg protein^−1^.

### Mitochondrial respiratory chain complex I and IV enzyme activity

Mitochondrial ETC complex I and complex IV activities were determined in tissue lysates following established protocols [11, 21–23]. All samples were analyzed in duplicates on the Cary UV-vis spectrophotometer (Varion, Inc., Palo Alto, CA).

### Superoxide dismutase and catalase enzyme activity

Muscle total superoxide dismutase (Mn-SOD and Cu/Zn-SOD) activity was determined in muscle lysates by measuring the kinetic consumption of superoxide radical (O_2_^−^) by SOD in a competitive reaction with cytochrome *c*, as previously described [20]. Absorption was recorded at 550 nm and was observed every 15 s for 2 min at 37 °C. One unit (U) of SOD activity was defined as the amount of enzyme that caused a 50 % inhibition of the reduction of cytochrome *c*. Total SOD activity was expressed in U.mg of protein^−1^. In a separate cuvette, the same sample was analyzed under identical conditions in the presence of 0.2 M KCN (pH 8.5–9.5), a potent inhibitor of cytosolic Cu/Zn-SOD [24], for determination of mitochondrial Mn-SOD activity. Cu/Zn-SOD activity was approximated by subtracting Mn-SOD activity from total SOD activity. Both Mn-SOD and Cu/Zn-SOD activity were expressed in U.mg protein^−1^. Catalase activity was determined by measuring the kinetic decomposition of H_2_O_2_ as previously described [25]. Catalase activity was measured by combining 960 μL of K_2_HPO_4_ buffer (50 mM with 50 mM EDTA and 0.01 % Triton X-100, pH 7.2–7.4) with 30 μL of muscle homogenate. Ten microliters of H_2_O_2_ (1 M) was added to the cuvette and mixed by inversion to initiate the reaction. Absorbance was measured at 240 nm every 15 s for 2 min. Catalase activity was calculated and reported in μmol · min^−1^ · mg protein^−1^. All samples were analyzed in duplicates on the Cary UV-vis spectrophotometer (Varion, Inc., Palo Alto, CA).

### Caspase-3 and caspase-9 enzyme activity

Caspase-3 and caspase-9 enzyme activity was measured using fluorometric protease assays caspase-3/CPP32 and caspase-9/Mch6, respectively (Biovision, Mountain View, CA) according to manufacturer’s instructions. Briefly, the assays are based on the detection of cleavage of the substrate DEVD-AFC (AFC: 7-amino-4-trifluoromethyl coumarin) by caspase-3 and LEHD-AFC (AFC: 7-amino-4-trifluoromethyl coumarin) by caspase-9. Uncleaved DEVD-AFC and LEHD-AFC fluoresce at *λ*_max_ = 400 nm, upon cleavage of the respective substrate by caspase-3 or caspase-9, free AFC emits a yellow-green fluorescence (*λ*_max_ = 505 nm), which was quantified using a fluorescence microplate reader (Tecan Safire, MTX Lab Systems, Inc., Vienna, VA). Results were expressed as raw fluorescence units per milligram of cytosolic protein.

The article "Exercise-induced mitochondrial p53 repairs mtDNA mutations in mutator mice" was retracted in 2021. Reason: duplicated images.

### Apoptosis cell death detection ELISA

Apoptotic DNA fragmentation was quantified in the skeletal muscle (*quadriceps femoris*), heart, primary hematopoietic stem cells, and primary satellite cells by measuring the amount of cytosolic mono- and oligo-nucleosomes using a Cell Death detection ELISA^PLUS^ assay (Roche Applied Science, Laval, QC) as previously described [11]. Briefly, wells were coated with a monoclonal anti-histone antibody and incubated with homogenates. Nucleosomes were centrifuged at 100,000*g* followed by binding to the anti-histone antibody followed by the addition of anti-DNA-peroxidase antibody that binds to the DNA associated with the histones. The amount of peroxidase retained in the immunocomplex was determined spectrophotometrically with ABTS (2,2′-azino-bis[3-ethylbenzthiazoline-6-sulphonic acid]) as a substrate. Results were expressed as arbitrary OD units normalized to micrograms of cytosolic protein.

### Quantification of mtDNA mutations

mtDNA mutations were quantified by the error-resistant single molecule approach [26]. Briefly, skeletal muscle (*quadriceps femoris*) DNA was subjected to limiting dilution long-range PCR, where each positive PCR reaction was initiated by a single mtDNA molecule. PCR was designed to amplify essentially the entire mitochondrial genome using high-fidelity Phusion DNA polymerase, (New England Biolabs). Three to 9 amplified molecules were obtained per animal. Each amplified molecule was sequenced in its entirety using barcoded Illumina next generation sequencing approach at a local core facility. Mutations were identified by comparing each molecule’s sequence to the standard C57Bl/6J mtDNA sequence (GenBank EF108336). Only 100 % mutations were considered, which guaranteed the exclusion of artifacts [26]. Mutant fractions were calculated by dividing the total number of mutations by the number of nucleotides sequenced per animal.

### p53 base excision repair activity assay

An in vitro fluorescence-based DNA primer p53 repair activity assay was employed as previously described [27], with minor modifications. This assay utilized a double-stranded deoxyoligomers containing sequences identical to the first 40 nucleotides of the mtDNA replication origin as the primer-template substrate, with the 3′ end of the primer contained self-designed mismatch point mutation in the last three nucleotides (Additional file 1: Table S2). The 5′ and 3′ ends of the primer were chemically linked to a Black Hole Quencher^®^-1 and 6-carboxyfluorescein (FAM-1™) flourophore, respectively (Integrated DNA Technology^®^, Toronto, ON). The premise of this assay is that, in the absence of proofreading capacity of mitochondrial polymerase gamma, primer extension requires the excision of the unpaired nucleotides by the 3′→5′ exonuclease activity which in turn will be detected as an increase in fluorescence over time. The 20 μL reaction mixtures containing 50 mM Tris–HCl (pH 7.5), 5 mM MgCl_2_, 1 mM DTT, 100 μg/mL of BSA, 3′-end-FAM1™ primer-template substrate, 50 μM each of dATP, dCTP, dGTP, and dTTP, and 40 μg of WT, PolG-SED, and PolG-END skeletal muscle (*quadriceps femoris*) mitochondrial extracts were incubated at 37 °C for 40 min with data collection at the end using iCycler IQ™ real-time PCR detection system (BioRad, Mississauga, ON). To assess the requirement of p53 as an accessory mtDNA mismatch point mutation repair protein, p53 repair activity assay was also carried out in (i) PolG-END skeletal muscle mitochondrial extract after p53 immunodepletion and (ii) PolG-SED skeletal muscle mitochondrial extract with addition of recombinant human p53 (BD Biosciences, Mississauga, ON).

The article "Exercise-induced mitochondrial p53 repairs mtDNA mutations in mutator mice" was retracted in 2021. Reason: duplicated images.

### Statistics

All molecular indices between the groups (WT, PolG-SED, PolG-END, PolG-p53 MKO-SED, and PolG-p53 MKO-END mice) were analyzed using two-tailed Student’s *t* test. The log-rank test was used to test for significant differences in life span distribution between groups. Statistical significance was established at a *P* ≤ 0.05. Data are presented as mean ± standard error of the mean (SEM).

## Results and discussion

### Endurance exercise confers phenotypic protection, reduces mtDNA mutations, and attenuates oxidative damage in PolG mice

Aged tissues display stochastic accumulation of mtDNA mutations that likely perpetuate respiratory chain deficiency and greater reactive oxygen species (ROS)-mediated damage [28]. To evaluate the underlying protective mechanism of exercise on mitochondrial redox status and mtDNA integrity, we profiled “terminally differentiated” (skeletal muscle and heart) and “proliferative” (Lin− Sca-1+ c-Kit + population enriched for hematopoietic stem and progenitor cells, “HSC’ and c-met+, satellite cells, “SC”) compartments of littermate wild-type (WT), sedentary PolG (PolG-SED), and forced-endurance exercised PolG (PolG-END) mice. As shown previously [11], and now confirmed in an independent cohort of mice utilized in this study, exercise rescued progeroid aging (Additional file 1: Figure S1A), increased life span (Additional file 1: Figure S1B), and reduced mtDNA mutations (Fig. 1a) in PolG mice.

The article "Exercise-induced mitochondrial p53 repairs mtDNA mutations in mutator mice" was retracted in 2021. Reason: duplicated images.

**Fig. 1:** Endurance exercise reduces random mtDNA somatic mutations, attenuates mitochondrial ROS-mediated oxidative damage, mitigates telomere shortening, and reduces nuclear accumulation of p53 in mtDNA mutator mice. **a** Random mtDNA somatic mutation rate (per 1000 nucleotides of mtDNA) in muscle (*quadriceps femoris*) WT, PolG-SED, and PolG-END mice (*n* = 4–5/group). **b** H_2_O_2_ production rate in muscle mitochondrial fractions of WT, PolG-SED, and PolG-END (*n* = 5–7/group). Complex I and II substrates: P/M, pyruvate/malate and SUC, succinate (5 mM each), respectively. Complex I and III inhibitors: ROT, rotenone, and AA, antimycin A (0.5 μM each), respectively. **c** Protein carbonyls (*PC*) content in muscle (*tibialis anterior*) and heart mitochondrial fractions of WT, PolG-SED, and PolG-END (*n* = 5–7/group). **d** SOD2 and catalase enzyme activity in the muscle (*quadriceps femoris*) and heart of WT, PolG-SED, and PolG-END (*n* = 7/group). **e** Average telomere length ratios in the heart, hematopoietic stem and progenitor cells (*HSC*), and satellite cells (*SC*) of WT, PolG-SED, and PolG-END (*n* = 6–8/group). **f** Representative blots of nuclear p53 content (~53 kDa) in the muscle (*quadriceps femoris*) and heart of WT, PolG-SED, and PolG-END (*n* = 5–8/group). Histone H2B (~14 kDa) was used as a nuclear loading control. (PolG-SED vs. both WT and PolG-END) = *P < 0.05, **P < 0.01; (PolG-END vs. WT) = ^†^ *P* < 0.05. *Error bars* represent SEM. *AU* arbitrary units

Initial characterization of PolG mice showed absence of increased oxidative damage despite significant accumulation of mtDNA point mutations [4, 29]. We evaluated the presence of oxidative modifications and found no difference in protein carbonyls (PC) and 4-hydroxy-2-nonenal (4-HNE) content in the muscle, heart, and SC homogenates of PolG-SED vs. WT (Additional file 1: Figure S1C). We surmised that since the absence of oxidative damage in the PolG tissues is due to cell-to-cell variability, and that any one modification would be lower than the detectable limit in whole tissue homogenates [4, 29], we measured oxidative damage in mitochondrial fractions—the primary source of cellular ROS. Indeed, mitochondria from these tissues demonstrated a substantial increase in H_2_O_2_ production, along with elevated PC and 4-HNE content (Fig. 1b, c, and Additional file 1: Figure S1C, D, and F). These observations are consistent with recent studies reporting higher PC levels in heart mitochondria of PolG mice [30] and increased mitochondrial H_2_O_2_ production in vivo using mitochondria-targeted mass spectrometry probe MitoB [31]. This higher oxidative damage is also congruent with reduced superoxide dismutase 2 (SOD2) and catalase content and activity in PolG-SED vs. WT (Fig. 1d and Additional file 1: Figure S1E). We hypothesize that the combination of lower antioxidant capacity, coupled with elevated ROS production in PolG-SED mitochondria exacerbates the accumulation of mtDNA mutations. Consistent with this notion, Vermulst et al. reported a significant reduction in the frequency of mtDNA mutations in the heart tissue of transgenic animals that over-expressed human catalase (CAT), a ROS scavenger, to mitochondria vs. age-matched (28 months old) wild-type mice [32]. We observed that exercise normalized mitochondrial H_2_O_2_ production (Fig. 1b and Additional file 1: Figure S1D), and markers of oxidative damage (Fig. 1c and Additional file 1: Figure S1F) in PolG-END to WT levels and increased SOD2 and catalase content and activity (Fig. 1d and Additional file 1: Figure S1E). Together, our data suggest that exercise reduces mtDNA point mutations, at least in part, via the up-regulation of cellular antioxidant capacity that subsequently serves to attenuate ROS levels.

The article "Exercise-induced mitochondrial p53 repairs mtDNA mutations in mutator mice" was retracted in 2021. Reason: duplicated images.

### Endurance exercise diminishes telomere erosion and down-regulates aberrant p53 signaling and pathological levels of apoptosis in PolG mice

Sustained intrinsic accumulation of oxidative damage has been implicated in telomere erosion that drives age-related tissue degeneration [1]. In agreement with this, we observed shorter telomeres in the heart, HSC, and SC from PolG-SED vs. WT (Fig. 1e). Genomic instability due to telomere shortening activates tumor suppressor protein p53-mediated senescence/apoptotic signaling cascades [1]. Accordingly, nuclear p53 abundance in the muscle, heart, and SC of PolG-SED was enhanced (Fig. 1f), concomitantly with higher expression levels of the p53-responsive senescence genes: p21^WAF1^, p16^INK4A^, and GADD45B (Additional file 1: Figure S1G) vs. WT. Mitochondrial dysfunction in PolG mice is associated with pathological systemic apoptosis [4, 11], and consistent with these observations, we found higher DNA fragmentation (Fig. 2a) and caspase-3/9 activity (Additional file 1: Figure S2A and B) in PolG-SED mice. Interestingly, exercise abrogated telomere shortening (Fig. 1e), reduced p53 nuclear accumulation (Fig. 1f), normalized the expression of p53-responsive senescence genes (Additional file 1: Figure S1G), and reduced pathological levels of apoptosis in PolG-END (Fig. 2a, and Additional file 1: Figure S2A and B).

**Fig. 2:** Endurance exercise prevents dysregulated mitochondrial-induced apoptosis, reduces nuclear p53-mediated repression of PGC-1α, induces PGC-1α regulated gene networks, restores mtDNA copy number, and normalizes mitochondrial morphology in mtDNA mutator mice. **a** Nuclear DNA fragmentation (apoptotic index) in the heart, HSC, and SC of WT, PolG-SED, and PolG-END (*n* = 7–10/group). **b** ChIP assay showing reduced p53 enrichment of PGC-1α promoter (positions −954/−564) with exercise in the muscle and heart of WT, PolG-SED, and PolG-END (*n* = 6/group). **c** Gene expression of PGC-1α and its downstream targets in muscle (*quadriceps femoris*), **d** mtDNA copy number normalized to nuclear β-globin gene in the muscle (*soleus*) and heart, and **e** representative electron micrographs of myofibers (*quadriceps femoris*) and cardiomyocytes (heart) from WT, PolG-SED, and PolG-END mice (*n* = 4–7/group). *Asterisk* (PolG-SED vs. both WT and PolG-END): *P < 0.05, **P < 0.01, ***P < 0.001. *Error bars* represent SEM. *AU* arbitrary units

The article "Exercise-induced mitochondrial p53 repairs mtDNA mutations in mutator mice" was retracted in 2021. Reason: duplicated images.

### Endurance exercise mitigates mitochondrial dysfunction via reduction in nuclear p53 that represses PGC-1α

A causal role of mitochondrial-induced oxidative stress and telomere erosion, secondary to mtDNA mutations, suggests a direct link between p53 activation and mitochondrial dysfunction [5]. Increasing the expression of PGC-1α, a potent regulator of mitochondrial biogenesis, positively regulates the expression of antioxidants [33] and has been touted to attenuate aging-associated sarcopenia and metabolic dysfunction [34]. This prompted us to investigate whether activation of p53-mediated senescence signaling attenuates PGC-1α-triggered gene programming. We conducted in silico promoter analysis that identified putative p53 binding elements in the PGC-1α promoter. These promoter regions were then cloned into a pGL4 luciferase reporter vector and transfected into *p53* ^*+/+*^ and *p53* ^*−/−*^ mouse embryonic fibroblasts (MEFs). A significant repression of PGC-1α-pGL4 reporter activity was observed in the *p53* ^*+/+*^ relative to *p53* ^*−/−*^ MEFs (Additional file 1: Figure S2C). These results are consistent with a recent study showing that nuclear p53 can directly repress PGC-1α expression and promote mitochondrial dysfunction [5]. To further test our hypothesis, we next performed an anti-p53 chromatin immunoprecipitation assay that showed physical enrichment of nuclear p53 at the PGC-1α promoter of PolG-SED vs. WT mice (Fig. 2b). Together, these data suggest that ROS-induced cellular damage prompts the nuclear accumulation of p53, which in turn activates p53-responsive senescence genes while simultaneously repressing the pro-metabolic activity of PGC-1α.

qPCR analyses of the PolG-SED muscle, heart, HSC and SC confirmed lower expression of PGC-1α and strong repression of its metabolic networks, including oxidative phosphorylation, mitochondrial function, gluconeogenesis, and fatty acid metabolism vs. WT (Fig. 2c, and Additional file 1: Figure S2D–G, and Table S1). Additionally, PolG-SED mice tissues and stem cells have reduced mtDNA copy number (Fig. 2D and Additional file 1: Figure S3A), lower mitochondrial complex I and complex IV enzyme activity (Additional file 1: Figure S3B), reduced mitochondrial electron transport chain subunits protein content (Additional file 1: Figure S3C–I), and accumulation of swollen, pleomorphic, oversized mitochondria (Fig. 2e). Endurance exercise decreased binding of p53 to the PGC-1α promoter (Fig. 2b), and this effect was accompanied by the maintenance of mtDNA copy number, increased expression of PGC-1α and its downstream metabolic network, enhanced mitochondrial oxidative capacity, and restoration of mitochondrial structural integrity in PolG-END (Fig. 2c–e, and Additional file 1: Figures S2D–G, Figure S3A–I, and Table S1). These observations collectively imply that accumulating mtDNA mutations in PolG-SED mice lead to an increase in ROS generation that (i) promotes mitochondrial dysfunction and telomere damage and (ii) subsequently triggers p53-regulated senescence pathways, thereby potentiating the loss of somatic and stem cells via apoptosis. In contrast, exercise reduced mtDNA mutations and maintained the cellular energy and redox homeostasis thereby circumventing telomere erosion culminating in the inhibition of accelerated systemic aging characteristic of PolG mice [3, 4].

The article "Exercise-induced mitochondrial p53 repairs mtDNA mutations in mutator mice" was retracted in 2021. Reason: duplicated images.

### Endurance exercise-mediated repair of mtDNA mutations is p53-dependent

POLG1 is the sole mitochondrial polymerase essential for mtDNA replication and repair via its 3′→5′ exonuclease activity [35]. Since exercise reduced mtDNA mutations in PolG mice, which lack proofreading capacity of POLG1, this raised an intriguing possibility that exercise recruited a POLG1-independent mtDNA repair pathway(s) [11]. We found that despite elevated p53 nuclear abundance in PolG-SED, the total p53 content in the muscle, heart, and SC homogenates of all groups was unaltered (Additional file 1: Figure S3J). This indicated that a basal pool of p53 is maintained intra-cellularly, with the distribution of p53 between the different subcellular compartments dependant on the cellular stress milieu [27]. In vitro studies show that in response to intra- and extra-cellular insults such as ROS, p53 translocates into the mitochondria where it interacts with the mtDNA and POLG1 [27]. Biochemical analysis of p53 has revealed an inherent 3′→5′ exonuclease activity that helps p53 promote and maintain mitochondrial genomic stability by executing base excision repair on damaged mtDNA [36]. The role of mitochondrial p53 in the context of aging remains hitherto unknown. Collectively, these observations led us to hypothesize that in the presence of an error-prone POLG1, mitochondrial p53 will function as an accessory fidelity-enhancing component of the mtDNA replication machinery in PolG mice.

The article "Exercise-induced mitochondrial p53 repairs mtDNA mutations in mutator mice" was retracted in 2021. Reason: duplicated images.

To test our hypothesis, we first assessed the submitochondrial localization of p53 in skeletal muscle of WT mice. Subfractionation of skeletal muscle mitochondria indicated that mitochondrial p53 was primarily localized in the mitochondrial matrix (Fig. 3a). Next, we measured the mitochondrial abundance of p53 in our experimental groups. Unlike PolG-SED, in PolG-END mice, p53 preferentially resided in the mitochondria vs. nuclei of muscle and heart (Figs. 1f and 3b). To ascertain whether mitochondrial ROS levels regulated p53 compartmentalization, we treated primary fibroblasts with rotenone, a complex I inhibitor known to increase mitochondrial ROS, and observed a rapid increase in mitochondrial p53 content at lower dosages without a concomitant increase in nuclear p53 (Additional file 1: Figure S4A). Intriguingly, with increasing rotenone concentrations, we measured an increase in nuclear p53 abundance (Additional file 1: Figure S4A) and expression of its downstream targets (p16^INK4A^ and p21^WAF1^; Additional file 1: Figure S4B), along with a concomitant reduction in mitochondrial p53 content (Additional file 1: Figure S4A), and mtDNA copy number (Additional file 1: Figure S4C). The increase in nuclear p53 paralleled the decrease in PGC-1α mRNA expression (Additional file 1: Figure S5A), further supporting the inhibitory effects of p53 on PGC-1α. Furthermore, the up-regulation of rotenone-evoked nuclear p53 content was attenuated in fibroblasts pre-treated with a ROS scavenger, *N*-acetylcysteine (Additional file 1: Figure S5B), in tandem with higher PGC-1α mRNA expression (Additional file 1: Figure S5C). Thus, p53 preferentially shuttles into mitochondria in response to physiological ROS levels, which abrogates the negative regulation of PGC-1α as exerted by p53 residing in the nucleus. Next, we sought to elucidate if mitochondrial p53 interacted with POLG1 and Tfam in the mitochondrial matrix. We performed co-immunoprecipitation reactions and found that mitochondrial p53 formed a complex with POLG1 and Tfam complexed at mtDNA (Fig. 3c–e). The p53-POLG1-Tfam complex at mtDNA was higher in PolG-END vs. PolG-SED and WT (Fig. 3c–e). These observations are consistent with a recent study reporting p53 translocation to of p53 to the mitochondria and subsequent formation of p53-Tfam-mtDNA complex in skeletal muscle of WT mice in response to an acute bout of endurance exercise [37]. These results led us to conclude that the preferential subcellular localization of p53 to mitochondria vs. nuclear compartment is a “universal” exercise-induced phenomenon and likely plays a role in mediating beneficial effects of endurance exercise on improving mitochondrial content/function and ameliorating dysfunction.

The article "Exercise-induced mitochondrial p53 repairs mtDNA mutations in mutator mice" was retracted in 2021. Reason: duplicated images.

**Fig. 3:** Endurance exercise increases the abundance of p53 in mitochondrial matrix where it interacts with mtDNA in a complex with POLG1 and Tfam in mtDNA mutator mice. **a** Mitochondrial p53 is primarily localized in the matrix. Muscle mitochondria were subfractionated into outer mitochondrial membrane (OMM), intermembrane space (IMS), inner mitochondrial membrane (IMM), and matrix (Mx) fractions, and these fractions were immunoblotted for the compartment-specific proteins TOMM22 (~16 kDa), cytochrome *c* (~14 kDa), COX-IV (~17 kDa), and CS (~45 kDa), respectively, and also for p53 (~53 kDa) and Tfam (~24 kDa). Representative blots of **b** mitochondrial p53 content (~53 kDa) in the muscle and heart of WT, PolG-SED, PolG-END (*n =* 6–8/group), **c** p53 co-immunoprecipitation (*IP*) followed by immunoblotting (*IB*) for mitochondrial transcription factor A (Tfam; ~24 kDa) to assess mitochondrial p53-Tfam complex content in muscle and heart mitochondria from WT, PolG-SED, PolG-END (*n =* 4–5/group), and **d** p53 co-*IP* followed by *IB* for POLG1 (~140 kDa) to assess mitochondrial p53-POLG1 complex content in muscle and heart mitochondria from WT, PolG-SED, and PolG-END (*n =* 6–8/group). VDAC (~32 kDa) was used as a mitochondrial loading control. **e** p53-POLG1-Tfam complex is bound to mtDNA (quantified using two independent mtDNA regions: COX-II and cytochrome *b*) in muscle mitochondrial fractions of WT, PolG-SED, and PolG-END mice (*n =* 4–6/group). A non-specific IgG antibody was used as negative control antibody. *Asterisk* (PolG-SED vs. both WT and PolG-END): *P < 0.05, **P < 0.01; dagger (PolG-END vs. WT): ^†^ *P* < 0.05. *Error bars* represent SEM. *AU* arbitrary units

Since both PolG-SED and PolG-END mice have defective POLG1 proofreading capacity, we believe that the reduction in total mtDNA mutational burden in PolG-END mice (Fig. 1a) is mediated by mitochondrial p53 levels in response to endurance exercise. Hence, we sought to evaluate whether mitochondrial p53 can repair mtDNA mutations, independent of the proofreading capacity of POLG1. A fluorescence-based in vitro DNA primer extension-mutation repair assay displayed an efficient repair of double-stranded oligonucleotides, with artificially added mismatch point mutations, incubated with ex vivo muscle mitochondrial extract of PolG-END vs. PolG-SED (Fig. 4a). PolG-END mitochondria failed to repair these mutations upon p53 immunodepletion (Fig. 4b), while addition of recombinant p53 increased PolG-SED mitochondrial mutation repair efficiency (Additional file 1: Figure S6A). Clearly, mitochondrial p53 plays a vital role in the maintenance of mtDNA integrity in the presence of defective POLG1 in mutator mice.

The article "Exercise-induced mitochondrial p53 repairs mtDNA mutations in mutator mice" was retracted in 2021. Reason: duplicated images.

**Fig. 4:** Endurance exercise-mediated repair of mtDNA mutations is mitochondrial p53-dependent. **a** A fluorescence-based in vitro DNA primer extension-mutation repair assay in muscle mitochondrial extracts from WT, PolG-SED, and PolG-END (*n =* 6–8/group) to assess the excision of the unpaired artificial point mutations. **b** p53 immunodepletion prevents mutation repair in muscle mitochondrial extracts from PolG-END (*n =* 5/group). A non-specific IgG antibody was used as negative control antibody. **c** Endurance stress test time to exhaustion in four independent trials in WT, PolG-SED, PolG-END, PolG-p53 MKO-SED, and PolG-p53 MKO-END mice (*n =* 5–6/group). **d** Representative electron micrographs of myofibers (*quadriceps femoris*) from WT, PolG-SED, PolG-END, PolG-p53 MKO-SED, and PolG-p53 MKO-END (*n =* 4/group). **e** Random mtDNA somatic mutation rate (per 1000 nucleotides of mtDNA) in muscle (*quadriceps femoris*) WT, PolG-SED, PolG-END, PolG-p53 MKO-SED, and PolG-p53 MKO-END mice (*n =* 3–4/group). **f** mtDNA copy number in muscle mitochondria from PolG-SED, PolG-END, PolG-p53 MKO-SED, and PolG-p53 MKO-END mice (*n =* 4–5/group) relative to WT mice (*horizontal line*). **g** Cytochrome *c* oxidase (COX) activity in muscle from WT, PolG-SED, PolG-END, PolG-p53 MKO-SED, and PolG-p53 MKO-END mice (*n =* 4–5/group). *Asterisk* (PolG-SED vs. both WT and PolG-END): *P < 0.05, **P < 0.01, ***P < 0.001; dagger (PolG-p53 MKO-SED vs. PolG-SED OR PolG-p53 MKO-END vs. PolG-END): ^†^ *P* < 0.05; *closed circle* (PolG-END vs. PolG-SED): ●*P* < 0.05, ●●*P* < 0.01, ●●●*P* < 0.001. *Error bars* represent SEM. *AU* arbitrary units

However, to conclusively attribute causality to mitochondrial p53 in mediating mtDNA repair in vivo in response to endurance exercise, a “double genetically altered mutator mouse model” was needed where changes in mtDNA mutation burden can be assessed in a background of p53 over-expression or knockdown. It was unfeasible to generate PolG mice with over-expression of p53, as previous work has shown that mice engineered with hyperactive p53 alleles display show stem cell depletion and premature aging phenotype themselves [38]. On the other hand, whole-body p53 knockout mice die prematurely of cancer [39] and do not breed efficiently with heterozygous *PolgA* ^*+/D257A*^ mice, and thus could not be bred with PolG mice to efficiently study the effects of exercise. Hence, we created a new genetically modified mutator mouse with muscle-specific p53 deletion (PolG-p53 MKO). At basal levels, PolG-p53 MKO-SED mice demonstrated an accelerated progeriod phenotype and significant accumulation of random mtDNA mutations in muscle compared to PolG-SED mice (Fig. 4e and Additional file 1: Figure S6B). To our surprise, endurance exercise not only failed to reduce mtDNA point mutations but also did not rescue progeroid aging, sarcopenia, exercise intolerance, mitochondrial morphology anomalies, and deficits in mitochondrial content and function such as mtDNA copy number, mitochondrial electron transport chain protein content, and COX activity in skeletal muscle of PolG-p53 MKO mice (Fig. 4c–g and Additional file 1: Figure S6B–E). This suggests that the exercise-mediated repair of mtDNA mutations in vivo is dependent on mitochondrial p53 adjuvant repair capacity. Furthermore, unlike PolG-END, mitochondrial extracts from PolG-p53 MKO failed to repair mutations in vitro in the primer extension-mutation repair assay (Additional file 1: Figure S6F). Thus, exercise-induced maintenance of mtDNA stability is contingent on mitochondrially localized p53 and represents a viable therapy for pre-symptomatic patients carrying POLG1 exonuclease domain mutations known to cause pathology [35].

The article "Exercise-induced mitochondrial p53 repairs mtDNA mutations in mutator mice" was retracted in 2021. Reason: duplicated images.

## Conclusions

Here, we show that exercise promotes mitochondrial oxidative capacity and cellular redox dynamics via PGC-1α-mediated expression networks, thus preventing the accumulation of oxidative damage, abrogating genotoxic damage, and repressing apoptosis in mutator mice. Intriguingly, stress-mediated subcellular localization of the tumor suppressor protein p53 determines its pro- or anti-survival function and seems indispensible for the exercise-mediated mtDNA repair and mitochondrial biogenesis. The work summarized here opens up viable avenues of research in cancer biology where mitochondrial dysfunction and genomic instability have been implicated [1]. It will be of potential clinical interest to see if exercise-induced mitochondrial-targeted p53 might represent a therapeutic intervention for aging-associated pathologies such as insulin resistance, diabetes, and cardiovascular diseases, which manifest telomere shortening in conjunction with mitochondrial dysfunction [40, 41]. Indeed, while exercise and an active lifestyle are the most prominent therapies to reduce the incidence and pathogenicity of diabetes, insulin resistance, and cardiovascular diseases [42, 43], therapeutic modalities that promise to recapitulate some of the effects of exercise warrant further attention. The telomere–p53–PGC-1α axis provides a molecular basis of how telomere erosion and mitochondrial dysfunction can modulate systemic aging of tissues and stem cell compartments. Understanding the upstream signaling cascades and posttranslational modifications that promote mitochondrial localization of p53 may allow for the generation of pharmaceutical analogs, novel therapeutic strategies to antagonize mitochondrial genomic decay, and cellular senescence in age-associated pathologies.

The article "Exercise-induced mitochondrial p53 repairs mtDNA mutations in mutator mice" was retracted in 2021. Reason: duplicated images.

## Additional file

Additional file 1: Figure S1. Endurance exercise confers complete phenotype protection, suppresses early mortality, mitigates mitochondrial ROS-mediated oxidative damage, increases cellular antioxidant capacity, and 4 prevents cellular senescencmutator mice. **Figure S2.** Endurance exercise prevents dysregulated mitochondrial-induced apoptosis and reduces nuclear p53-mediated repression of PGC-1α and promotes mitochondrial biogenesis in mutator mice. **Figure S3.** Endurance exercise promotes systemic mitochondrial biogenesis in mtDNA mutator mice. **Figure S4.** Magnitude of mitochondrial ROS (physiological vs. pathological) regulates p53 subcellular localization. **Figure S5.** Pre-treatment with exogenous antioxidant preferentially shuttles p53 to mitochondria in response to stress. **Figure S6.** Endurance exercise-mediated attenuation of sarcopenia, increase in endurance capacity, skeletal muscle mitochondrial biogenesis, and repair of muscle mtDNA mutations is p53 dependent. **Table S1.** WT, PolG-SED, and PolG-END Skeletal Muscle Microarray IPA-GO Analysis. **Table S2.** Real-time PCR primer sequences. (PDF 1601 kb)

## Abbreviations

4-HNE: 4-hydroxy-2-nonenal
ALAS: 5-aminolevulinate synthase
ATPase 6: complex V subunit ATPase 6
COX-I: cytochrome *c* oxidase subunit-I
COX-II: cytochrome *c* oxidase subunit-II
COX-IV: cytochrome *c* oxidase subunit-IV
END: endurance exercise
ERRα: estrogen-related receptor alpha
GADD45B: growth arrest and DNA-damage-inducible, beta
H_2_O_2_: hydrogen peroxide
HSC: hematopoietic stem and progenitor cells
MEF: mouse embryonic fibroblasts
MKO: muscle-specific knockout
mtDNA: mitochondrial DNA
ND1: complex I NADH dehydrogenase subunit 1
NRF1: nuclear respiratory factor 1
p16^INK4A^: cyclin-dependent kinase inhibitor 2A
p21^WAF1^: cyclin-dependent kinase inhibitor 1A
p53: tumor suppressor protein 53
PC: protein carbonyls
PGC-1α: peroxisome proliferator-activated receptor gamma co-activator 1 alpha
PolG: polymerase gamma mutator mice
POLG1: mitochondrial polymerase gamma
ROS: reactive oxygen species
SC: satellite cells
SED: sedentary
SOD1: superoxide dismutase 1 (cytosolic; Cu/Zn-SOD)
SOD2: superoxide dismutase 2 (mitochondrial; Mn-SOD)
TFAM: mitochondrial transcription factor A
VDAC: voltage-dependent anion channel
WT: wild-type mice
